# Poisson XLindley Distribution for Count Data: Statistical and Reliability Properties with Estimation Techniques and Inference

**DOI:** 10.1155/2022/6503670

**Published:** 2022-04-13

**Authors:** Muhammad Ahsan-ul-Haq, Afrah Al-Bossly, Mahmoud El-Morshedy, Mohamed S. Eliwa

**Affiliations:** ^1^College of Statistical and Actuarial Sciences, University of the Punjab, Lahore, Pakistan; ^2^Department of Mathematics, College of Science and Humanities in Al-Kharj, Prince Sattam Bin Abdulaziz University, Al-Kharj 11942, Saudi Arabia; ^3^Department of Mathematics, Faculty of Science, Mansoura University, Mansoura 35516, Egypt; ^4^Department of Statistics and Operation Research, College of Science, Qassim University, P.O. Box 6644, Buraydah 51482, Saudi Arabia; ^5^Department of Statistics and Computer Science, Faculty of Science, Mansoura University, Mansoura 35516, Egypt

## Abstract

In this study, a new one-parameter count distribution is proposed by combining Poisson and XLindley distributions. Some of its statistical and reliability properties including order statistics, hazard rate function, reversed hazard rate function, mode, factorial moments, probability generating function, moment generating function, index of dispersion, Shannon entropy, Mills ratio, mean residual life function, and associated measures are investigated. All these properties can be expressed in explicit forms. It is found that the new probability mass function can be utilized to model positively skewed data with leptokurtic shape. Moreover, the new discrete distribution is considered a proper tool to model equi- and over-dispersed phenomena with increasing hazard rate function. The distribution parameter is estimated by different six estimation approaches, and the behavior of these methods is explored using the Monte Carlo simulation. Finally, two applications to real life are presented herein to illustrate the flexibility of the new model.

## 1. Introduction 

Researchers obtain a multitude of probability distributions for analyzing the various forms of data sets from diverse sectors, such as health, transportation, engineering, astronomy, and agriculture. Various well-known approaches are used to introduce new probability distributions. Some famous approaches, such as compounding technique and T-X family, give a very effective way to generalize a common parametric family of distributions to fit data sets and those classical distributions do not sufficiently fit. In some practical fields, count data may be generated/observed, and to model such data, discrete probability distributions were proposed based on different approaches such as survival discretization, Poisson mixture, and compound models. For example, Greenwood and Yule [1] compound Poisson and negative binomial distributions by considering the rate parameter in the Poisson distribution. Mahmoudi and Zakerzadeh [2] extended the Poisson–Lindley distribution and revealed that their generalized distribution is more flexible in evaluating count data. Zamani and Ismail [3] introduced a novel compound distribution by combining a negative binomial distribution with a one-parameter Lindley distribution that provides a better fit for count data. Rashid [4] introduced a count data model that combines the negative binomial and Kumaraswamy distributions and used it for modeling biological data sets. Some more discrete distributions are Poisson–Ishita distribution by Hassan et al. [5]; Poisson–Ailamujia distribution by Hassan et al. [6]; Poisson Xgamma distribution by Para et al. [7]; Poisson quasi-Lindley distribution by Grine and Zeghdoudi [8]; discrete Gompertz-G family by Eliwa et al. [9]; discrete extension to three-parameter Lindley model by Eliwa et al. [10]; two-parameter exponentiated discrete Lindley distribution by El-Morshedy et al. [11]; Eliwa and El-Morshedy [12]; discrete Burr–Hatke distribution by El-Morshedy et al. [13]; discrete Weibull Marshall–Olkin family by Gillariose et al. [14]; and discrete Ramos–Louzada model by Eldeeb et al. [15].

The XLindley (XL) distribution was introduced for the analysis of lifetime data (see [16]). Let *X* be a random variable following the XL distribution with the probability density function:

(1) $$\begin{array}{c} f\left(x\right)=\frac{\alpha^{2}\left(2+\alpha +x\right)e^{-\alpha x}}{{\left(1+\alpha \right)}^{2}};x>0,\alpha >0. \end{array}$$

Since there is a need for a more flexible model for modeling statistical data, in this study, we proposed a flexible discrete distribution by compounding Poisson and XL distributions. The proposed model is named the “Poisson-XL” distribution. The reported distribution strength lies in the capacity to describe equi- and over-dispersed data. Furthermore, it can be used as a suitable statistical tool to model positively skewed data with leptokurtic shape. One more advantage to Poisson-XL model is that its statistical and reliability characterization can be expressed in closed forms, which make this model have multi-benefits in regression and time-series analysis.

The study is organized as follows.  Section 2 is devoted to the derivation of Poisson-XL distribution and its shape analysis. Some statistical properties are derived in Section 3. Some reliability measures are derived in Section 4. The parameter is estimated in Section 5.  Section 6 is based on the applications of the proposed distribution. In the end, we concluded this study in Section 7.

## 2. Synthesis of the Poisson-XL Model

If *X|λ* follows Poisson(*λ*) where *λ* is itself a random variable following XL distribution with parameter *α*, then determining the distribution that results from marginalizing over *λ* will be known as a compound of Poisson distribution with that of XL distribution, which is denoted by the PXL model.

**Theorem 1 .**

The probability mass function of a compound of PXL distribution is given as follows:

(2) $$\begin{array}{c} P\left(x\right)=P_{PXL\;D}\left(X=x,\alpha \right)=\frac{\alpha^{2}\left(x+\alpha^{2}+3\left(1+\alpha \right)\right)}{{\left(1+\alpha \right)}^{4+x}};x=0,1,2,\ldots ,\alpha >0. \end{array}$$

**Proof**

The probability mass function of a compound of Poisson(*λ*) with *XL*(*α*) can be formulated as follows:

(3) $$\begin{array}{c} P\left(X=\lambda ,\alpha \right)=\int_{0}^{\infty }p_{1}\left(x|\lambda \right)f_{1}\left(x,\lambda \right)\text{d}\lambda . \end{array}$$

Then:

(4) $$\begin{array}{c} P\left(X=\lambda ,\alpha \right)=\int_{0}^{\infty }\frac{e^{-\lambda }\lambda^{x}}{x!}\frac{\alpha^{2}\left(2+\alpha +\lambda \right)e^{-\alpha \lambda }}{{\left(1+\alpha \right)}^{2}}\text{d}\lambda ,\\ =\frac{\alpha^{2}}{{\left(1+\alpha \right)}^{2}x!}\int_{0}^{\infty }\lambda^{x}\left(2+\alpha +\lambda \right)e^{-\lambda \left(\alpha +1\right)}\text{d}\lambda ,\\ =\frac{\alpha^{2}\left(x+\alpha^{2}+3\left(1+\alpha \right)\right)}{{\left(1+\alpha \right)}^{4+x}}, \end{array}$$

where *x*=0,1,2,…,  and *α* > 0.  Figure 1 shows the probability mass function (PMF) plots of the proposed distribution for various values of parameter *α*.

According to Figure 1, it is noted that the PMF can be either unimodal or decreasing-shaped. Further, it can be utilized as a probability tool to discuss right-skewed data. The corresponding cumulative distribution function (CDF) to equation (2) can be expressed as follows:

(5) $$\begin{array}{c} F\left(X=x,\alpha \right)=\overset{x}{\underset{y=0}{\sum }}\frac{\alpha^{2}\left(y+\alpha^{2}+3\left(1+\alpha \right)\right)}{{\left(1+\alpha \right)}^{4+y}}=1-\frac{1}{{\left(1+\alpha \right)}^{4+x}}\left\{1+\alpha \left(x+4+\alpha \left(3+\alpha \right)\right)\right\}. \end{array}$$

where *x*=0,1,2,…,  and *α* > 0. Let *x*_1:*n*_, *x*_2:*n*_, *x*_3:*n*_,…, *x*_*n*:*n*_ be the order statistics of a random sample from the PXL distribution. The cumulative distribution function of *i*th order statistics for an integer value of *x* is given as follows:

(6) $$\begin{array}{c} F_{i:n}\left(x;\alpha \right)=\overset{n}{\underset{m=i}{\sum }}\left(\begin{array}{c} n\\ m \end{array}\right){\left[F_{i}\left(x;\alpha \right)\right]}^{m}{\left[1-F_{i}\left(x;\alpha \right)\right]}^{n-m}\\ =\overset{n}{\underset{m=i}{\sum }}\overset{n-m}{\underset{j=0}{\sum }}\Psi_{\left(k\right)}^{\left(n,m\right)}{\left[F_{i}\left(x;\alpha \right)\right]}^{m+j}\\ =\overset{n}{\underset{m=i}{\sum }}\overset{n-m}{\underset{j=0}{\sum }}\Psi_{\left(k\right)}^{\left(n,m\right)}F_{i}\left(x;\alpha ,m+j\right), \end{array}$$

where$\Psi_{\left(k\right)}^{\left(n,m\right)}={\left(-1\right)}^{j}\left(\begin{array}{c} n\\ m \end{array}\right)\left(\begin{array}{c} n-m\\ j \end{array}\right)$ and *F*_*i*_(*x*; *α*, *m*+*j*)=[1 − {1+*α*(*x*+4+*α*(3+*α*))}/(1+*α*)^4+*x*^]^*m*+*j*^ represent the CDF of the exponentiated PXL distribution with power *m*+*j*. The corresponding PMF to equation (2) is given as follows:

(7) $$\begin{array}{c} f_{i:n}\left(x;\alpha \right)=F_{i:n}\left(x;\alpha \right)-F_{i:n}\left(x-1;\alpha \right)\\ =\overset{n}{\underset{m=i}{\sum }}\overset{n-m}{\underset{j=0}{\sum }}\Psi_{\left(k\right)}^{\left(n,m\right)}f_{i}\left(x;\alpha ,m+j\right), \end{array}$$

where *f*_*i*_(*x*; *α*, *m*+*j*) represents the PMF of the exponentiated PXL distribution with power parameter *m*+*j*. Thus, the *p*th moments of *X*_*i*:*n*_ can be written as follows:

(8) $$\begin{array}{c} E\left(X_{i:n}^{p}\right)=\overset{\infty }{\underset{x=0}{\sum }}\overset{n}{\underset{m=i}{\sum }}\overset{n-m}{\underset{j=0}{\sum }}\Psi_{\left(k\right)}^{\left(n,m\right)}x^{p}f_{i}\left(x;\alpha ,m+j\right). \end{array}$$

## 3. Statistical Properties

### 3.1. Mode

To get and study the mode of the PXL model with its characterization, we should derive the first and second derivatives to the PMF with respect to *x*, where:

(9) $$\begin{array}{c} \frac{d}{dx}\left(P\left(X=\lambda ,\alpha \right)\right)=\frac{\alpha^{2}-\alpha^{2}\log\left(1+\alpha \right)\left(x+\alpha^{2}+3\left(\alpha +1\right)\right)}{{\left(1+\alpha \right)}^{4+x}},\\ \frac{{\text{d}}^{2}}{\text{d}x^{2}}\left(P\left(X=\lambda ,\alpha \right)\right)=-\frac{2\alpha^{2}\log\left(1+\alpha \right)+{\left(\log\left(1+\alpha \right)\right)}^{2}\left(x+\alpha^{2}+3\left(\alpha +1\right)\right)}{{\left(1+\alpha \right)}^{4+x}}, \end{array}$$

and when *d*/*dx*(*P*(*X*=*λ*, *α*))=0, the solution is as follows:

(10) $$\begin{array}{c} \hat{x}=\frac{1}{\log\left(1+\alpha \right)}-\left(\alpha^{2}+3\alpha +3\right),\\ \frac{d^{2}}{dx^{2}}\left(P{\left(X=\lambda ,\alpha \right)}_{x=\hat{x}}\right)=-\frac{2\alpha^{2}\log\left(1+\alpha \right)}{{\left(1+\alpha \right)}^{1/\log\left(1+\alpha \right)-\alpha^{2}-3\alpha +1}}<0. \end{array}$$

For $\alpha ,\hat{x}>0,$ the mode is a unique critical point, in which *P*(*X*=*λ*, *α*) is maximum and *P*(*X*=*λ*, *α*) is concave, but if $\hat{x}<0$ the density function is decreasing of *x*.

### 3.2. Factorial Moments

The *r*th factorial moment around the origin of the PXL distribution can be obtained as follows:

(11) $$\begin{array}{c} \mu_{\left(r\right)}^{\prime }=\mu_{\left(r\right)}^{\prime }=E\left[E\left(X^{\left(r\right)}|\lambda \right)\right]=\int_{0}^{\infty }\left(\overset{\infty }{\underset{x=0}{\sum }}x^{\left(r\right)}\frac{e^{-\lambda }\lambda^{x}}{x!}\right)\frac{\alpha^{2}\left(2+\alpha +\lambda \right)e^{-\alpha \lambda }}{{\left(1+\alpha \right)}^{2}}\text{d}\lambda , \end{array}$$

where *X*^(*r*)^=*X*(*X* − 1)(*X* − 2) … (*X* − *r*+1), and then:

(12) $$\begin{array}{c} \mu_{\left(r\right)}^{\prime }=\frac{\alpha^{2}}{{\left(1+\alpha \right)}^{2}}\int_{0}^{\infty }\lambda^{r}\left(\overset{\infty }{\underset{x=r}{\sum }}\frac{e^{-\lambda }\lambda^{x-r}}{\left(x-r\right)!}\right)\left(2+\alpha +\lambda \right)e^{-\alpha \lambda }\text{d}\lambda , \end{array}$$

and assuming *y*=*x* − *r*, we get the following:

(13) $$\begin{array}{c} \mu_{\left(r\right)}^{\prime }=\frac{\alpha^{2}}{{\left(1+\alpha \right)}^{2}}\int_{0}^{\infty }\lambda^{r}\left(\overset{\infty }{\underset{y=0}{\sum }}\frac{e^{-\lambda }\lambda^{y}}{y!}\right)\left(2+\alpha +\lambda \right)e^{-\alpha \lambda }\text{d}\lambda ,\\ \mu_{\left(r\right)}^{\prime }=\frac{\alpha^{2}}{{\left(1+\alpha \right)}^{2}}\left[\left(2+\alpha \right)\int_{0}^{\infty }\lambda^{r}e^{-\alpha \lambda }\text{d}\lambda +\int_{0}^{\infty }\lambda^{r+1}e^{-\alpha \lambda }\text{d}\lambda \right]\\ =\left[\frac{\alpha \left(\alpha +2\right)+\left(r+1\right)}{{\left(1+\alpha \right)}^{2}}\right]. \end{array}$$

### 3.3. Probability Generating Function (PGF)

**Theorem 2 .**

If *X* has PXL(*X*; *α*), then PGF *G*_*x*_(*Z*) can be formulated as follows:

(14) $$\begin{array}{c} G_{x}\left(Z\right)=\frac{\alpha^{2}}{{\left(1+\alpha \right)}^{3}}\left\{\frac{z+\left(1+\alpha -z\right)\left(\alpha^{2}+3\left(1+\alpha \right)\right)}{{\left(1+\alpha -z\right)}^{2}}\right\};\alpha >0. \end{array}$$

**Proof**

The PGF can be obtained as follows:

(15) $$\begin{array}{c} G_{x}\left(Z\right)=\overset{\infty }{\underset{x=0}{\sum }}Z^{x}p\left(x\right)=\overset{\infty }{\underset{x=0}{\sum }}Z^{x}\frac{\alpha^{2}\left(x+\alpha^{2}+3\left(1+\alpha \right)\right)}{{\left(1+\alpha \right)}^{4+x}}\\ =\frac{\alpha^{2}}{{\left(1+\alpha \right)}^{4}}\overset{\infty }{\underset{x=0}{\sum }}Z^{x}\frac{\left(x+\alpha^{2}+3\left(1+\alpha \right)\right)}{{\left(1+\alpha \right)}^{x}}\\ =\frac{\alpha^{2}}{{\left(1+\alpha \right)}^{4}}\left\{\overset{\infty }{\underset{x=0}{\sum }}\frac{xZ^{x}}{{\left(1+\alpha \right)}^{x}}+\left(\alpha^{2}+3\left(1+\alpha \right)\right)\overset{\infty }{\underset{x=0}{\sum }}\frac{Z^{x}}{{\left(1+\alpha \right)}^{x}}\right\}\\ =\frac{\alpha^{2}}{{\left(1+\alpha \right)}^{4}}\left\{\frac{z}{1+\alpha }{\left(\frac{1+\alpha }{1+\alpha -z}\right)}^{2}+\left(\alpha^{2}+3\left(1+\alpha \right)\right)\left(\frac{1+\alpha }{1+\alpha -z}\right)\right\}\\ =\frac{\alpha^{2}}{{\left(1+\alpha \right)}^{3}}\left\{\frac{z}{{\left(1+\alpha -z\right)}^{2}}+\frac{\left(\alpha^{2}+3\left(1+\alpha \right)\right)}{\left(1+\alpha -z\right)}\right\}. \end{array}$$

### 3.4. Moment Generating Function (MGF)

**Theorem 3 .**

If *X* has PXL(*X*; *α*), then the MGF can be expressed as follows:

(16) $$\begin{array}{c} M_{x}\left(t\right)=\frac{\alpha^{2}}{{\left(1+\alpha \right)}^{3}}\left\{\frac{e^{t}+\left(1+\alpha -e^{t}\right)\left(\alpha^{2}+3\left(1+\alpha \right)\right)}{{\left(1+\alpha -e^{t}\right)}^{2}}\right\};\alpha >0. \end{array}$$

**Proof**

The moments around the origin can be obtained as follows:

(17) $$\begin{array}{c} M_{x}\left(t\right)=\overset{\infty }{\underset{x=0}{\sum }}e^{tx}P\left(x\right)=\overset{\infty }{\underset{x=0}{\sum }}e^{tx}\frac{\alpha^{2}\left(x+\alpha^{2}+3\left(1+\alpha \right)\right)}{{\left(1+\alpha \right)}^{4+x}}\\ =\frac{\alpha^{2}}{{\left(1+\alpha \right)}^{4}}\left\{\overset{\infty }{\underset{x=0}{\sum }}\frac{xe^{tx}}{{\left(1+\alpha \right)}^{x}}+\left(\alpha^{2}+3\left(1+\alpha \right)\right)\overset{\infty }{\underset{x=0}{\sum }}\frac{e^{tx}}{{\left(1+\alpha \right)}^{x}}\right\}\\ =\frac{\alpha^{2}}{{\left(1+\alpha \right)}^{4}}\left\{\frac{e^{t}}{1+\alpha }{\left(\frac{1+\alpha }{1+\alpha -e^{t}}\right)}^{2}+\left(\alpha^{2}+3\left(1+\alpha \right)\right)\left(\frac{1+\alpha }{1+\alpha -e^{t}}\right)\right\}. \end{array}$$

Then:

(18) $$\begin{array}{c} M_{x}\left(t\right)=\frac{\alpha^{2}}{{\left(1+\alpha \right)}^{3}}\left\{\frac{e^{t}}{{\left(1+\alpha -e^{t}\right)}^{2}}+\frac{\left(\alpha^{2}+3\left(1+\alpha \right)\right)}{\left(1+\alpha -e^{t}\right)}\right\}. \end{array}$$

The first four ordinary moments of *X* are as follows:

(19) $$\begin{array}{c} \mu_{1}^{\prime }=\frac{\alpha^{2}+2\alpha +2}{\alpha {\left(1+\alpha \right)}^{2}},\\ \mu_{2}^{\prime }=\frac{\alpha^{3}+4\alpha^{2}+6\alpha +6}{\alpha^{2}{\left(1+\alpha \right)}^{2}},\\ \mu_{3}^{\prime }=\frac{\alpha^{4}+8\alpha^{3}+20\alpha^{2}+30\alpha +24,}{\alpha^{3}{\left(1+\alpha \right)}^{2}}\\ \mu_{4}^{\prime }=\frac{\left[\alpha^{5}+16\alpha^{4}+66\alpha^{3}+138\alpha^{2}+192\alpha +120\right]}{\alpha^{4}{\left(1+\alpha \right)}^{2}}, \end{array}$$

whereas the first four moments around the mean of *X* are as follows:

(20) $$\begin{array}{c} \mu_{1}=\frac{\alpha^{2}+2\alpha +2}{\alpha {\left(1+\alpha \right)}^{2}},\\ \mu_{2}=\frac{\alpha^{5}+5\alpha^{4}+11\alpha^{3}+14\alpha^{2}+10\alpha +2}{\alpha^{2}{\left(1+\alpha \right)}^{4}},\\ \mu_{3}=\frac{\alpha^{8}+9\alpha^{7}+36\alpha^{6}+87\alpha^{5}+141\alpha^{4}+152\alpha^{3}+98\alpha^{2}+30\alpha +4}{\alpha^{3}{\left(1+\alpha \right)}^{6}},\\ \mu_{4}=\frac{1}{\alpha^{4}{\left(1+\alpha \right)}^{8}}\left\{\begin{array}{c} \alpha^{11}+18\alpha^{10}+127\alpha^{9}+515\alpha^{8}+1395\alpha^{7}+2692\alpha^{6}\\ +3747\alpha^{5}+3678\alpha^{4}+2430\alpha^{3}+1010\alpha^{2}+240\alpha +24 \end{array}\right\}. \end{array}$$

Based on the rth moments, the index of dispersion index (DI) can be expressed as follows:

(21) $$\begin{array}{c} DI=\frac{Var\left(X\right)}{E\left(X\right)}=\frac{\alpha^{5}+5\alpha^{4}+11\alpha^{3}+14\alpha^{2}+10\alpha +2}{\alpha^{4}+2\alpha^{3}+3\alpha^{2}+2\alpha +2}. \end{array}$$

Further, the skewness and kurtosis can be derived in closed forms, where:

(22) $$\begin{array}{c} S=\frac{\mu_{3}-3\mu_{2}\mu_{1}+2{\left(\mu_{1}\right)}^{3}}{{\left(\mu_{2}\right)}^{1.5}},\\ K=\frac{\mu_{4}-4\mu_{3}\mu_{1}+6\mu_{2}{\left(\mu_{1}\right)}^{2}-3{\left(\mu_{1}\right)}^{4}}{{\left(\mu_{2}\right)}^{2}}. \end{array}$$

The summary measure, mean, variance, moments, and DI are presented in Table 1. The PXL model can be used to model equi- and over-dispersed data.

The plots of coefficient of skewness and kurtosis are shown in Figure 2. The skewness and kurtosis monotonically increase for higher values of *α*. Moreover, the PXL model can be used as a probability tool for modeling positively skewed data with leptokurtic shape.

### 3.5. Shannon Entropy

The Shannon entropy is a measurable physical property that is most associated with a state of disorder, randomness, or uncertainty. The term and the concept are used in diverse fields, from classical thermodynamics, where it was first recognized, to the microscopic description of nature in statistical physics, and to the principles of information theory. The Shannon entropy of the random variable *X* can be expressed as follows:

(23) $$\begin{array}{c} H\left(x\right)=-\overset{\infty }{\underset{x=0}{\sum }}P\left(X=x;\alpha \right)\log\left[P\left(X=x;\alpha \right)\right], \end{array}$$

and then:

(24) $$\begin{array}{c} H\left(x\right)=-\overset{\infty }{\underset{x=0}{\sum }}\frac{\alpha^{2}\left(x+\alpha^{2}+3\left(1+\alpha \right)\right)}{{\left(1+\alpha \right)}^{4+x}}\left\{\log\left(\alpha^{2}\right)+\log\left(x+\alpha^{2}+3\alpha +3\right)-\left(4+x\right)\log\left(1+\alpha \right)\right\}\\ =-\log\left(\alpha^{2}\right)-\frac{\alpha^{2}}{{\left(1+\alpha \right)}^{4}}\overset{\infty }{\underset{x=0}{\sum }}\frac{\left(x+\alpha^{2}+3\left(1+\alpha \right)\right)\log\left(x+\alpha^{2}+3\left(1+\alpha \right)\right)}{{\left(1+\alpha \right)}^{x}}\\ +\frac{\log\left(1+\alpha \right)\alpha^{2}}{{\left(1+\alpha \right)}^{4}}\overset{\infty }{\underset{x=0}{\sum }}\frac{\left(x+\alpha^{2}+3\left(1+\alpha \right)\right)\left(4+x\right)}{{\left(1+\alpha \right)}^{x}}\\ =-\log\left(\alpha^{2}\right)+\frac{\alpha^{2}{\text{HurwitzLerchPhi}}^{\left(0,1,0\right)}\left[1/1+\alpha ,-1,\alpha^{2}+3\left(1+\alpha \right)\right]}{{\left(1+\alpha \right)}^{4}}\\ +\frac{\left(2+10\alpha +23\alpha^{2}+28\alpha^{3}+17\alpha^{4}+4\alpha^{5}\right)\log\left(1+\alpha \right)}{\alpha {\left(1+\alpha \right)}^{4}}. \end{array}$$

For more details around HurwitzLerchPhi (0, 1, 0) function “Lerch transcendent,” see https://mathworld.wolfram.com/LerchTranscendent.html. Some entropy values of PXL distribution in terms of the parameter (*α*) are presented in Table 2. It is noticed that the Shannon entropy shows a monotonically decreasing pattern and it proceeds to zero when *α* increased.

## 4. Reliability Characteristics of the PXL Distribution

### 4.1. Reversed (Hazard) Rate Function and Mills Ratio

The corresponding survival function (SF) to equation (5) can be expressed as follows:

(25) $$\begin{array}{c} S\left(x;\alpha \right)=\frac{1}{{\left(1+\alpha \right)}^{3+x}}\left\{1+\alpha \left(x+4+\alpha \left(3+\alpha \right)\right)\right\};x=0,1,2,3,\ldots . \end{array}$$

The hazard rate function (HRF) of the random variable *X* can be defined as *h*(*x*)=*P*(*X*=*x*; *α*)/*S*(*x* − 1; *α*). Then, the HRF of the PXL distribution can be formulated as follows:

(26) $$\begin{array}{c} h\left(x\right)=\frac{\alpha^{2}\left(x+\alpha^{2}+3\left(1+\alpha \right)\right)}{\left(1+\alpha \right)\left\{1+\alpha \left(x+\alpha^{2}+3\left(1+\alpha \right)\right)\right\}}. \end{array}$$

It is easy to see that the limiting behavior HRF at the upper limit is $\underset{x⟶\infty }{\lim}h\left(x\right)=\left(\alpha /1+\alpha \right)$. As a result, the parameter *α* may be regarded as a strict upper bound on the HRF, which is a key feature of lifetime probability distributions. Few discrete distributions contain parameters that can be readily interpretable in terms of failure rate functions. The geometric distribution is an exception, although in this instance the HRF is constant. In Proposition 1, we proved that the PXL distribution always allows for increasing failure rates.

**Proposition 1 .**

The HRF of the PXL distribution is increasing.

**Proof**

According to Glaser (1980) and from the PMF of the PXL distribution:

(27) $$\begin{array}{c} \eta \left(x\right)=-\frac{P^{\prime }\left(x\right)}{P\left(x\right)}=\frac{-1+\log\left(1+\alpha \right)\left(x+\alpha^{2}+3\left(1+\alpha \right)\right)}{x+\alpha^{2}+3\left(1+\alpha \right)}, \end{array}$$

and it follows that:

(28) $$\begin{array}{c} \eta^{\prime }\left(x\right)=\frac{1}{{\left(x+\alpha^{2}+3\left(1+\alpha \right)\right)}^{2}}>0, \end{array}$$

∀*x*, *α* > 0, implying that *h*(*x*) is increasing.  Figure 3 illustrates some plots of the PXL model based on various values of the model parameter.

The reverse hazard rate of the PXL distribution is as follows:

(29) $$\begin{array}{c} r^{*}\left(x\right)=\frac{P\left(x\right)}{F\left(x\right)}=\frac{\alpha^{2}\left(x+\alpha^{2}+3\left(1+\alpha \right)\right)}{{\left(1+\alpha \right)}^{4+x}-\left\{1+\alpha \left(x+4+\alpha \left(3+\alpha \right)\right)\right\}}, \end{array}$$

whereas the second rate of failure and Mills ratio can be expressed, respectively, as follows:

(30) $$\begin{array}{c} r^{**}\left(x\right)=\log\left[\frac{S\left(x\right)}{S\left(x+1\right)}\right]=\;\log\left[\frac{\left(1+\alpha \right)\left\{1+\alpha \left(x+\alpha^{2}+3+3\alpha \right)\right\}}{\left\{1+\alpha \left(x+\alpha^{2}+4+3\alpha \right)\right\}}\right],\\ M=\frac{S\left(x\right)}{p\left(x\right)}=\frac{\left(1+\right)\left\{1+\alpha \left(x+4+\alpha \left(3+\alpha \right)\right)\right\}}{\alpha^{2}\left(x+\alpha^{2}+3\left(1+\alpha \right)\right)}. \end{array}$$

### 4.2. Mean Residual Life

For the random variable *X*, the mean residual life or the mean remaining lifetime (MRL) is the expected remaining life of *X* − *t*, given that the item has survived to time *i*. Thus, the MRL concept can be used effectively in stochastic ageing and dependence for reliability. The unconditional mean of the distribution, *E*(*X*), is a special case of mean residual life for *i*=0. For a discrete random variable, the MRL function is defined as follows:

(31) $$\begin{array}{c} \varepsilon \left(i\right)=E\left(X-i|X\geq i\right)=\frac{1}{1-F\left(i-1,\alpha \right)}\overset{w}{\underset{j=i+1}{\sum }}\left[1-F\left(j-1,\alpha \right)\right];i\in {\mathbb{N}}_{0}, \end{array}$$

where *ℕ*_0_={0, 1, 2,…, *w*} and 0 < *w* < *∞*. Let *X* have the PXL random variable, and then, the MRL is defined as follows:

(32) $$\begin{array}{c} \varepsilon \left(i\right)=\frac{{\left(1+\alpha \right)}^{3+i}}{\left\{1+\alpha \left(i+3+\alpha \left(3+\alpha \right)\right)\right\}}\overset{w}{\underset{j=i+1}{\sum }}\left[\frac{\left\{1+\alpha \left(j+3+\alpha \left(3+\alpha \right)\right)\right\}}{{\left(1+\alpha \right)}^{3+j}}\right]\\ =\frac{{\left(1+\alpha \right)}^{i}}{\left\{1+\alpha \left(i+3+\alpha \left(3+\alpha \right)\right)\right\}}\overset{w}{\underset{j=i+1}{\sum }}\left[\frac{\left\{1+\alpha \left(j+3+\alpha \left(3+\alpha \right)\right)\right\}}{{\left(1+\alpha \right)}^{j}}\right], \end{array}$$

and after simple algebra steps, we get the MRL in an explicit form as follows:

(33) $$\begin{array}{c} \varepsilon \left(i\right)=\frac{{\left(1+\alpha \right)}^{i}}{\left\{1+\alpha \left(i+3+\alpha \left(3+\alpha \right)\right)\right\}}\left\{\begin{array}{c} \left[1+\alpha \left(3+\alpha \left(3+\alpha \right)\right)\right]\\ \overset{w}{\underset{j=i+1}{\sum }}\frac{1}{{\left(1+\alpha \right)}^{j}}+\alpha \overset{w}{\underset{j=i+1}{\sum }}\frac{j}{{\left(1+\alpha \right)}^{j}} \end{array}\right\}\\ =\frac{1}{\left\{1+\alpha \left(i+3+\alpha \left(3+\alpha \right)\right)\right\}}\left\{\left[1+\alpha \left(3+\alpha \left(3+\alpha \right)\right)\right]\frac{1}{\alpha }+\alpha \left(i+\frac{1+\alpha }{\alpha }\right)\right\}\\ =\frac{\left\{1+\alpha \left(i\alpha +4+\alpha \left(4+\alpha \right)\right)\right\}}{\alpha \left\{1+\alpha \left(i+3+\alpha \left(3+\alpha \right)\right)\right\}}. \end{array}$$

## 5. Various Estimation Techniques

This section is based on parameter estimation of the PXL distribution using different estimation methods. The considered methods are maximum likelihood, moment, Anderson darling, Cramér–von Mises, ordinary least squares, and weighted least squares.

### 5.1. Maximum-Likelihood Estimation (MLE)

Suppose *x*=(*x*_1_, *x*_2_, *x*_3_,…, *x*_*n*_) be a random sample of size “*n*” from the PXL distribution. Then, the log-likelihood (*L*) function is given as follows:

(34) $$\begin{array}{c} L=2n\;\log\;\alpha +\overset{n}{\underset{i=1}{\sum }}\log\left(x_{i}+\alpha^{2}+3\left(1+\alpha \right)\right)-\overset{n}{\underset{i=1}{\sum }}\left(4+x_{i}\right)\log\left(1+\alpha \right). \end{array}$$

Partially differentiating with respect to *α*, we get the following:

(35) $$\begin{array}{c} \frac{\partial L}{\partial \alpha }=\frac{2n}{\alpha }+\overset{n}{\underset{i=1}{\sum }}\frac{2\alpha +3}{\left(x_{i}+\alpha^{2}+3\left(1+\alpha \right)\right)}-\overset{n}{\underset{i=1}{\sum }}\frac{\left(4+x_{i}\right)}{\left(1+\alpha \right)}. \end{array}$$

Since we cannot get a close form to equation (15), a numerical procedure should be used to solve this equation numerically to get the maximum-likelihood estimator.

### 5.2. Method of Moment Estimation (MOME)

Based on the MOME approach for estimating the parameter, the sample and population means should be derived. So, to get the estimator of the PXL model, the solution of the following nonlinear equation provides the estimate of *α*, where:

(36) $$\begin{array}{c} \bar{x}=\frac{\alpha^{2}+2\alpha +2}{\alpha {\left(1+\alpha \right)}^{2}}. \end{array}$$

### 5.3. Anderson–Darling Estimation (ADE)

The ADE is based on the difference in empirical and fitted CDF. The ADE of *α* follows by minimizing:

(37) $$\begin{array}{c} \text{ADE}\left(\alpha \right)=-n-\frac{1}{n}\overset{n}{\underset{i=1}{\sum }}\left(2i-1\right)\left[\begin{array}{c} \log\left[1-\frac{1}{{\left(1+\alpha \right)}^{4+i}}\left\{1+\alpha \left(x_{i:n}+4+\alpha \left(3+\alpha \right)\right)\right\}\right]\\ +\log\left[\frac{1}{{\left(1+\alpha \right)}^{4+i}}\left\{1+\alpha \left(x_{i:n}+4+\alpha \left(3+\alpha \right)\right)\right\}\right] \end{array}\right], \end{array}$$

with respect to *α*.

### 5.4. Cramér–von Mises Estimation (CVME)

The CVME is based on the difference between empirical and fitted CDF. The CVME of *α* follows by minimizing:

(38) $$\begin{array}{c} \text{CVME}\left(\alpha \right)=\frac{1}{12n}+\overset{n}{\underset{i=1}{\sum }}{\left[1-\frac{1}{{\left(1+\alpha \right)}^{4+i}}\left\{1+\alpha \left(x_{i:n}+4+\alpha \left(3+\alpha \right)\right)\right\}-\frac{2i-1}{2n}\right]}^{2}, \end{array}$$

with respect to *α*.

### 5.5. Ordinary Least-Squares and Weighted Least-Squares Estimation

Let *X*_*i*:*n*_ be the *i*th order statistics in a sample of size *n*. We adopt lower cases for sample values. It is well known that:

(39) $$\begin{array}{c} E\left[F\left(X_{i:n}\right)\right]=\frac{i}{1+n}\text{and}V\left[F\left(X_{i:n}\right)\right]=\frac{i\left(n-i+1\right)}{{\left(n+1\right)}^{2}\left(n+2\right)}. \end{array}$$

Thus, the least-squares estimate (LSE) of *α*, say $\hat{\alpha }$, can be derived by minimizing:

(40) $$\begin{array}{c} \text{LSE}\left(\alpha \right)=\overset{n}{\underset{i=1}{\sum }}{\left[1-\frac{1}{{\left(1+\alpha \right)}^{4+i}}\left\{1+\alpha \left(x_{i:n}+4+\alpha \left(3+\alpha \right)\right)\right\}-\frac{i}{n+1}\right]}^{2}, \end{array}$$

with respect to *α*. The weighted least-squares estimate (WLSE) of *α*, say $\hat{\alpha }$, can be determined by minimizing:

(41) $$\begin{array}{c} \text{WLSE}\left(\alpha \right)=\overset{n}{\underset{i=1}{\sum }}\frac{{\left(n+1\right)}^{2}\left(n+2\right)}{i\left(n-i+1\right)}{\left[1-\frac{1}{{\left(1+\alpha \right)}^{4+i}}\left\{1+\alpha \left(x_{i:n}+4+\alpha \left(3+\alpha \right)\right)\right\}-\frac{i}{n+1}\right]}^{2}, \end{array}$$

with respect to *α*.

## 6. Simulation

To assess the accuracy of the six estimators described previously, we conducted a comprehensive simulation study. We used the PXL distribution to generate samples with *n*=25, 50, 100, 200, and 500 and then calculated the average values (AVEs) of the MLE, MOME, LSE, WLSE, CVME, and ADE to get the mean square errors (MSEs), average absolute biases (ABBs), and mean relative errors (MREs) for *α*=0.3, 0.5, 1.0, and 1.5. The ABBs, MREs, and MSEs are given as follows:

(42) $$\begin{array}{c} \text{ABBs}=\frac{\sum_{i=1}^{N}\left|\hat{\alpha }-\alpha \right|}{N},\\ \text{MREs}=\frac{\sum_{i=1}^{N}\left|\hat{\alpha }-\alpha \right|/a}{N},\\ \text{MSE}=\frac{\sum_{i=1}^{N}{\left(\hat{\alpha }-\alpha \right)}^{2}}{N}. \end{array}$$

We ran the simulation 5000 times to derive these metrics from the prior values for all estimation methods. The findings in Tables 3–6 were obtained using the R software's optim-CG function. The findings show that as the sample size *n* increased, the AVEs became closer to the real values of *α*. Furthermore, when *n* increases, the ABBs, MREs, and MSEs for all estimators decreased.

## 7. Applications

In this section, the flexibility of the PXL distribution is proposed based on two distinctive real data sets. The first data set is the biological experiment data on the European corn borer [17], which is shown in Table 7. The investigator counts the number of borers per hill of corn in an experiment conducted randomly on 8 hills in 15 replications. The mean, variance, and index of dispersion values of *X* are 1.4833, 3.193, and 2.1526, respectively. Since distribution is over-dispersed, we can use PXL distribution.

The second data set shows the number of mammalian cytogenetic dosimetry lesions produced by streptogramin (NSC-45383) exposure in rabbit lymphoblasts of −70 3 bc g/kg [18]. The second data set is shown in Table 8. The mean, variance, and index of dispersion values of *X* are 0.54, 0.8312, and 1.5392, respectively.

Some competitive models such as the discrete Bilal (DB) by Altun et al. [19]; discrete Pareto (DPr) by Krishna and Pundir [20]; discrete Rayleigh (DR) by Roy [21]; discrete Burr–Hatke (DBH) by El-Morshedy et al. (2020); discrete inverted Topp–Leone (DITL) by Eldeeb et al. [22]; Poisson–Ailamujia (PA) by Hassan et al. [6]; and Poisson (Poi) distributions are used herein. To obtain the best model to analyze data sets I and II, some criteria should be used such as Akaike information criterion (AIC) and Bayesian information criterion (BIC) as well as −*L* as indicators of the relative quality of statistical models for the given set of data. These criteria assess the quality of each model with the other models given a set of data models. Moreover, the chi-square (*χ*^2^) test is used with its corresponding *p* value where the estimated probabilities under the null hypothesis are as follows:

(43) $$\begin{array}{c} {\hat{\alpha }}_{i}=\hat{P}\left(X=i\right)=\frac{\alpha^{2}\left(i+\alpha^{2}+3\left(1+\alpha \right)\right)}{{\left(1+\alpha \right)}^{4+i}};i=0,1,2,3,\ldots . \end{array}$$

The estimated expected frequencies are obtained as ${\hat{e}}_{i}=n{\hat{\alpha }}_{i}$. The results of the chi-square test are reported in Tables 7 and 8. Thus, we cannot reject the null hypothesis at the 5% level of significance and the PXL distribution is a good fit for these data sets.

For data set I, the PXL and PA work quite well for analyzing data set I, but the PXL is the best, and Figure 4 supports our empirical results, which are listed in Table 7. For data set II, the PXL, DBH, and DITL work quite well for analyzing data set II, but the PXL is the best, and Figure 5 supports our empirical results, which are reported in Table 8. Since one of the major aims of this study is to get the best estimators for the data sets I and II, several estimation techniques have been derived for this purpose. Tables 9 and 10 report the different estimators for data sets I and II based on various estimation techniques.

It is noted that MLE and MOME approaches work quite well in analyzing data set I, but the MLE method is the best for these data, whereas data set II can be discussed via the MLE and MOME techniques, but the MLE is the best.

## 8. Conclusion

In this study, a new one-parameter Poisson–XLindley (PXL) distribution has been proposed for modeling count data. Some distributional properties are derived and studied in detail. It was found that the properties of the PXL can be expressed in closed forms, which make it a proposer probability tool to establish regression and time-series model for discussing different types of data sets in various fields. The new probability mass function can be utilized to model positively skewed data with leptokurtic shape. Moreover, the PXL model can be used to model equi- and over-dispersed phenomena with increasing hazard rate function. Different estimation approaches have been used to estimate the model parameter. The behavior of these methods has been explored using the Monte Carlo simulation. Finally, two applications to real life have been discussed to illustrate the flexibility of the new discrete model.

## Figures and Tables

**Figure 1:** PMF plot of the PXL distribution.

**Figure 2:** Skewness and kurtosis of the PXL distribution.

**Figure 3:** HRF plots of the PXL distribution.

**Figure 4:** Fitted PMFs of all selected models for the first data set.

**Figure 5:** Fitted PMFs of all selected models for the second data set.

**Table 1:** Moments and DI of the PXL distribution.

*α*	Mean	Variance	DI	*E*(*X*^2^)	*E*(*X*^3^)	*E*(*X*^4^)
0.1	18.265	215.25	11.785	548.84	22486.0	1162376.9
0.2	8.4722	56.138	6.6261	127.92	2679.3	71386.3
0.5	2.8889	9.6543	3.3419	18.000	160.22	1847.3
0.7	1.9229	5.1317	2.6687	8.8292	58.293	502.48
1.0	1.2500	2.6875	2.1500	4.2500	20.750	133.25
1.5	0.7733	1.3486	1.7439	1.9467	6.9244	32.548
2.0	0.5556	0.8580	1.5444	1.1667	3.3889	13.000
2.5	0.4327	0.6177	1.4277	0.8049	2.0274	6.7216
3.0	0.3542	0.4787	1.3517	0.6042	1.3681	4.0579
3.5	0.2998	0.3893	1.2985	0.4792	0.9987	2.7111
4.0	0.2600	0.3274	1.2592	0.3950	0.7700	1.9438
4.5	0.2296	0.2822	1.2291	0.3349	0.6178	1.4671
5.0	0.2056	0.2477	1.2053	0.2900	0.5109	1.1513
7.0	0.1451	0.1661	1.1450	0.1872	0.2897	0.5602
10	0.1008	0.1110	1.1008	0.1212	0.1680	0.2825
50	0.0200	0.0204	1.0200	0.0208	0.0225	0.0259
100	0.0100	0.0101	1.0100	0.0102	0.0106	0.0114

**Table 2:** Shannon entropy of PXL distribution.

*α*	*H*(*x*)	*α*	*H*(*x*)	*α*	*H*(*x*)
0.1	3.88282	3.0	0.77819	6.5	0.45858
0.2	3.17056	3.5	0.70201	7.0	0.43522
0.5	2.21336	4.0	0.64144	7.5	0.41444
1.0	1.54538	4.5	0.59193	8.0	0.39582
1.5	1.21462	5.0	0.55056	8.5	0.37901
2.0	1.01384	5.5	0.51539	100	0.05611
2.5	0.87756	6.0	0.48506	500	0.01443

**Table 3:** Simulation results of PXL distribution for *α*=0.3.

*n*		MLE	MOME	ADE	CVME	OLSE	WLSE
25	AVEs	0.3342	0.3341	0.2907	0.2913	0.2912	0.2863
50		0.3296	0.3307	0.2886	0.2887	0.2887	0.2819
100		0.3279	0.3279	0.2876	0.2884	0.2881	0.2782
200		0.3264	0.3260	0.2874	0.2876	0.2876	0.2750
500		0.3257	0.3261	0.2875	0.2873	0.2872	0.2711

25	AABs	0.0342	0.0341	0.0093	0.0087	0.0088	0.0137
50		0.0296	0.0307	0.0114	0.0113	0.0113	0.0181
100		0.0279	0.0279	0.0124	0.0116	0.0119	0.0218
200		0.0264	0.0260	0.0126	0.0124	0.0124	0.0250
500		0.0257	0.0261	0.0125	0.0127	0.0128	0.0289

25	MREs	0.1626	0.0487	0.1168	0.1215	0.1234	0.1135
50		0.1252	0.0383	0.0874	0.0868	0.0879	0.0892
100		0.1041	0.0312	0.0657	0.0670	0.0663	0.0795
200		0.0912	0.0269	0.0531	0.0536	0.0533	0.0840
500		0.0859	0.0262	0.0445	0.0453	0.0456	0.0963

25	MSEs	0.0042	0.0041	0.0019	0.0021	0.0021	0.0017
50		0.0023	0.0024	0.0010	0.0010	0.0011	0.0011
100		0.0015	0.0015	0.0006	0.0006	0.0006	0.0008
200		0.0010	0.0010	0.0004	0.0004	0.0004	0.0008
500		0.0008	0.0008	0.0002	0.0003	0.0003	0.0009

**Table 4:** Simulation results of PXL distribution for *α*=0.5.

*n*		MLE	MOME	ADE	CVME	OLSE	WLSE
25	AVEs	0.6016	0.6006	0.4629	0.4614	0.4613	0.4387
50		0.5892	0.5914	0.4618	0.4588	0.4587	0.4282
100		0.5848	0.5860	0.4594	0.4577	0.4567	0.4164
200		0.5818	0.5834	0.4585	0.4564	0.4563	0.4065
500		0.5800	0.5811	0.4583	0.4566	0.4562	0.3950

25	AABs	0.1016	0.1006	0.0371	0.0386	0.0387	0.0613
50		0.0892	0.0914	0.0382	0.0412	0.0413	0.0718
100		0.0848	0.0860	0.0406	0.0423	0.0433	0.0836
200		0.0818	0.0834	0.0415	0.0436	0.0437	0.0935
500		0.0800	0.0811	0.0417	0.0434	0.0438	0.1050

25	MREs	0.2295	0.1153	0.1239	0.1244	0.1267	0.1379
50		0.1883	0.0965	0.0995	0.1035	0.1029	0.1454
100		0.1720	0.0874	0.0885	0.0914	0.0932	0.1672
200		0.1639	0.0835	0.0843	0.0886	0.0885	0.1870
500		0.1601	0.0811	0.0835	0.0868	0.0876	0.2099

25	MSEs	0.0234	0.0229	0.0056	0.0056	0.0058	0.0066
50		0.0136	0.0142	0.0035	0.0038	0.0038	0.0063
100		0.0100	0.0103	0.0027	0.0028	0.0029	0.0075
200		0.0080	0.0083	0.0022	0.0024	0.0024	0.0090
500		0.0069	0.0071	0.0019	0.0021	0.0021	0.0111

**Table 5:** Simulation results of PXL distribution for *α*=1.0.

*n*		MLE	MOME	ADE	CVME	OLSE	WLSE
25	AVEs	1.5469	1.5542	0.7898	0.7750	0.7717	0.6919
50		1.4910	1.4875	0.7875	0.7703	0.7708	0.6658
100		1.4592	1.4636	0.7857	0.7704	0.7685	0.6403
200		1.4475	1.4504	0.7865	0.7692	0.7683	0.6180
500		1.4408	1.4449	0.7851	0.7687	0.7681	0.5924

25	AABs	0.5469	0.5542	0.2102	0.2250	0.2283	0.3081
50		0.4910	0.4875	0.2125	0.2297	0.2292	0.3342
100		0.4592	0.4636	0.2143	0.2296	0.2315	0.3597
200		0.4475	0.4504	0.2135	0.2308	0.2317	0.3820
500		0.4408	0.4449	0.2149	0.2313	0.2319	0.4076

25	MREs	0.5529	0.5598	0.2107	0.2253	0.2285	0.3082
50		0.4919	0.4880	0.2125	0.2297	0.2292	0.3342
100		0.4592	0.4636	0.2143	0.2296	0.2315	0.3597
200		0.4475	0.4504	0.2135	0.2308	0.2317	0.3820
500		0.4408	0.4449	0.2149	0.2313	0.2319	0.4076

25	MSEs	0.4942	0.5189	0.0517	0.0574	0.0588	0.0994
50		0.3217	0.3169	0.0490	0.0561	0.0560	0.1137
100		0.2441	0.2499	0.0479	0.0543	0.0552	0.1303
200		0.2161	0.2190	0.0466	0.0541	0.0545	0.1463
500		0.2003	0.2043	0.0466	0.0538	0.0541	0.1663

**Table 6:** Simulation results of PXL distribution for *α*=1.5.

*n*	1.5	MLE	MOME	ADE	CVME	OLSE	WLSE
25	AVEs	3.3389	3.3799	0.9800	0.9544	0.9549	0.8498
50		3.0594	3.0595	0.9821	0.9535	0.9550	0.8133
100		2.9521	2.9474	0.9806	0.9534	0.9533	0.7817
200		2.8950	2.8800	0.9808	0.9522	0.9523	0.7540
500		2.8558	2.8612	0.9808	0.9518	0.9520	0.7209

25	AABs	1.8389	1.8799	0.5200	0.5456	0.5451	0.6502
50		1.5594	1.5595	0.5179	0.5465	0.5450	0.6867
100		1.4521	1.4474	0.5194	0.5466	0.5467	0.7183
200		1.3950	1.3800	0.5192	0.5478	0.5477	0.7460
500		1.3558	1.3612	0.5192	0.5482	0.5480	0.7791

25	MREs	1.2271	1.8812	0.3466	0.3637	0.3634	0.4335
50		1.0396	1.5595	0.3452	0.3643	0.3633	0.4578
100		0.9681	1.4474	0.3463	0.3644	0.3645	0.4789
200		0.9300	1.3800	0.3461	0.3652	0.3651	0.4973
500		0.9039	1.3612	0.3461	0.3655	0.3653	0.5194

25	MSEs	6.6135	7.2913	0.2765	0.3036	0.3032	0.4279
50		3.2428	3.2877	0.2713	0.3017	0.3001	0.4743
100		2.4086	2.4046	0.2714	0.3003	0.3005	0.5173
200		2.0792	2.0315	0.2704	0.3008	0.3007	0.5572
500		1.8857	1.9028	0.2698	0.3008	0.3006	0.6073

**Table 7:** Goodness of fit for data set I.

X	Observed frequency	Expected frequency							
		PXL	DB	Poi	DPr	DR	DBH	DITL	PA
0	43	47.1	32.7	27.2	64.5	15.9	68.1	52.2	39.6
1	35	29.2	39.6	40.4	20.1	36.2	22.0	30.4	33.7
2	17	17.8	24.3	30.0	9.7	34.6	10.5	14.1	21.5
3	11	10.7	12.5	14.8	5.6	21.0	6.0	7.5	12.2
4	5	6.3	6.0	5.5	3.7	8.9	3.8	4.4	6.5
5	4	3.7	2.7	1.6	2.6	2.7	2.5	2.8	3.3
6	1	2.2	1.2	0.4	1.9	0.6	1.7	1.9	1.7
7	2	1.3	0.5	0.1	1.5	0.1	1.3	1.3	0.8
8	2	1.7	0.4	0.0	10.4	0.0	4.2	5.4	0.7
Total	120	120	120	120	120	120	120	120	120
*α*	MLE	0.8661	0.2767	1.4833	1.1112	1.8743	0.8655	1.9840	0.6740
	S.E.	0.0822	0.1598	0.1111	0.1027	0.0874	0.0385	0.1832	0.0667

*χ* ^2^		1.8227	9.6428	21.898	36.243	60.179	25.142	6.9342	2.7097
Degree of freedom		4	4	3	4	3	3	4	4
*p* Value		0.7683	0.0468	<0.01	<0.01	<0.01	<0.01	<0.01	0.1394
−*L*		200.63	204.68	219.19	220.62	235.23	214.05	205.15	201.22
AIC		403.26	411.35	440.38	443.24	472.45	430.10	412.30	404.44
BIC		406.04	414.14	443.16	446.02	475.24	432.89	415.09	407.23

**Table 8:** Fitted PXL distribution and other competitor distributions to second data set.

X	Observed frequency	Expected frequency							
		PXL	DB	Poi	DPr	DR	DBH	DITL	PA
0	200	194.6	174.9	174.8	216.9	124.8	209.6	196.9	186.0
1	57	68.5	94.6	94.4	43.9	140.3	54.1	69.3	79.1
2	30	24.0	24.0	25.5	16.2	32.5	19.9	19.9	25.2
3	7	8.4	5.2	4.6	7.8	2.3	8.5	7.2	7.1
4≥	6	4.5	1.3	0.7	15.2	0.1	7.9	6.8	2.5
Total	300	300	300	300	300	300	300	300	300
*α*	MLE	2.0512	1.2332	0.5400	1.8518	0.9643	0.6030	3.7134	1.8519
	S.E.	0.1763	0.0551	0.0424	0.1124	0.0298	0.0376	0.2243	0.1639

*χ* ^2^		3.5508	26.547	30.431	22.663	96.650	6.4361	7.4422	9.3468
Degree of freedom		2	2	2	3	1	3	3	2
*p* Value		0.1694	<0.01	<0.01	<0.01	<0.01	0.0922	0.0591	<0.01
−*l*		299.31	311.74	314.23	312.94	371.12	301.70	302.76	302.41
AIC		600.63	625.48	630.45	627.88	744.23	605.41	607.53	606.83
BIC		604.33	629.18	634.16	631.59	747.94	609.11	611.23	610.53

**Table 9:** Estimation and goodness of fit for data set I.

Method ↓ Statistics⟶	*α*	*χ* ^2^	*p* Value
ADE	0.60116	14.49629	0.02456
CVME	0.59562	15.04585	0.01990
OLSE	0.59542	15.04585	0.01990
WLSE	0.50906	28.80345	<0.001
MOME	0.86747	1.839527	0.76524

**Table 10:** Estimation and goodness of fit for data set II.

Method ↓ Statistics⟶	*α*	*χ* ^2^	*p* Value
ADE	0.90250	96.36338	<0.001
CVME	0.87576	104.0459	<0.001
OLSE	0.87573	104.0550	<0.001
WLSE	0.67663	189.2819	<0.001
MOME	2.05081	3.558362	0.16666

## Data Availability

The datasets generated during the current study are available from the corresponding author on reasonable request.

## Appendix

- Plotting code for the probability mass function:
- DD2 <- 0 : 150
- PP2 <- *c* (0.6483923879*e* − 2, 0.8133981019*e* − 2, 0.9612187075*e* − 2, 0.1093116721*e* − 1, 0.1210273384*e* − 1, 0.1313793547*e* − 1, 0.1404710263*e* − 1, 0.1483989121*e* − 1, 0.1552532327*e* − 1, 0.1611182554*e* − 1, 0.1660726563*e* − 1, 0.1701898621*e* − 1, 0.1735383710*e* − 1, 0.1761820562*e* − 1, 0.1781804508*e* − 1, 0.1795890164*e* − 1, 0.1804593955*e* − 1, 0.1808396501*e* − 1, 0.1807744849*e* − 1, 0.1803054588*e* − 1, 0.1794711823*e* − 1, 0.1783075048*e* − 1, 0.1768476896*e* − 1, 0.1751225791*e* − 1, 0.1731607496*e* − 1, 0.1709886576*e* − 1, 0.1686307768*e* − 1, 0.1661097267*e* − 1, 0.1634463938*e* − 1, 0.1606600457*e* − 1, 0.1577684374*e* − 1, 0.1547879118*e* − 1, 0.1517334942*e* − 1, 0.1486189805*e* − 1, 0.1454570203*e* − 1, 0.1422591947*e* − 1, 0.1390360894*e* − 1, 0.1357973633*e* − 1, 0.1325518127*e* − 1, 0.1293074317*e* − 1, 0.1260714683*e* − 1, 0.1228504777*e* − 1, 0.1196503719*e* − 1, 0.1164764655*e* − 1, 0.1133335198*e* − 1, 0.1102257834*e* − 1, 0.1071570297*e* − 1, 0.1041305933*e* − 1, 0.1011494024*e* − 1, 0.9821601058*e* − 2, 0.9533262577*e* − 2, 0.9250113694*e* − 2, 0.8972314003*e* − 2, 0.8699996103*e* − 2, 0.8433267864*e* − 2, 0.8172214430*e* − 2, 0.7916900173*e* − 2, 0.7667370457*e* − 2, 0.7423653323*e* − 2, 0.7185761019*e* − 2, 0.6953691442*e* − 2, 0.6727429487*e* − 2, 0.6506948282*e* − 2, 0.6292210345*e* − 2, 0.6083168657*e* − 2, 0.5879767648*e* − 2, 0.5681944130*e* − 2, 0.5489628143*e* − 2, 0.5302743736*e* − 2, 0.5121209708*e* − 2, 0.4944940273*e* − 2, 0.4773845682*e* − 2, 0.4607832797*e* − 2, 0.4446805617*e* − 2, 0.4290665759*e* − 2, 0.4139312903*e* − 2, 0.3992645204*e* − 2, 0.3850559661*e* − 2, 0.3712952457*e* − 2, 0.3579719273*e* − 2, 0.3450755570*e* − 2, 0.3325956848*e* − 2, 0.3205218875*e* − 2, 0.3088437905*e* − 2, 0.2975510862*e* − 2, 0.2866335515*e* − 2, 0.2760810630*e* − 2, 0.2658836107*e* − 2, 0.2560313102*e* − 2, 0.2465144133*e* − 2, 0.2373233177*e* − 2, 0.2284485750*e* − 2, 0.2198808976*e* − 2, 0.2116111656*e* − 2, 0.2036304310*e* − 2, 0.1959299224*e* − 2, 0.1885010487*e* − 2, 0.1813354011*e* − 2, 0.1744247561*e* − 2, 0.1677610765*e* − 2, 0.1613365119*e* − 2, 0.1551434002*e* − 2, 0.1491742660*e* − 2, 0.1434218218*e* − 2, 0.1378789658*e* − 2, 0.1325387813*e* − 2, 0.1273945351*e* − 2, 0.1224396756*e* − 2, 0.1176678310*e* − 2, 0.1130728068*e* − 2, 0.1086485834*e* − 2, 0.1043893138*e* − 2, 0.1002893202*e* − 2, 0.9634309176*e* − 3, 0.9254528115*e* − 3, 0.8889070174*e* − 3, 0.8537432424*e* − 3, 0.8199127366*e* − 3, 0.7873682576*e* − 3, 0.7560640404*e* − 3, 0.7259557616*e* − 3, 0.6970005072*e* − 3, 0.6691567376*e* − 3, 0.6423842558*e* − 3, 0.6166441719*e* − 3, 0.5918988708*e* − 3, 0.5681119790*e* − 3, 0.5452483312*e* − 3, 0.5232739379*e* − 3, 0.5021559532*e* − 3, 0.4818626429*e* − 3, 0.4623633531*e* − 3, 0.4436284795*e* − 3, 0.4256294367*e* − 3, 0.4083386280*e* − 3, 0.3917294171*e* − 3, 0.3757760977*e* − 3, 0.3604538668*e* − 3, 0.3457387961*e* − 3, 0.3316078047*e* − 3, 0.3180386341*e* − 3, 0.3050098200*e* − 3, 0.2925006696*e* − 3, 0.2804912345*e* − 3, 0.2689622883*e* − 3, 0.2578953025*e* − 3, 0.2472724235*e* − 3, 0.2370764506*e* − 3, 0.2272908144*e* − 3, 0.2178995551*e* − 3, 0.2088873029*e* − 3)
- *y*range = *c* (0, 1)
- Segments (0, 0, 0, 0, lwd = 0)
- Plot (DD2, PP2, type = “*h*”, col = 4, main = expression (paste (alpha, “ = 0.05”)), cex.main = 1.0, *x*lab = “*x*”, *y*lab = “PMF”, lwd = 1, pch = 5)
- Points (DD2, PP2, col = 0); abline (*h* = 26, col = 2)
- Par (new = TRUE)
- Plot (DD2, PP2, type = “*p*”, col = 2, main = expression (paste (alpha, “ = 0.05”)), cex.main = 1.0, *x*lab = “*x*”, *y*lab = “PMF”, lwd = 1, pch = 1)
- Par (new = TRUE)
- Plotting code for the hazard rate function:
- DD1 <- 0 : 100
- PP1 <- *c*(0.7021604936*e* − 1, 0.8022130016*e* − 1, 0.8834586466*e* − 1, 0.9507445588*e* − 1, 0.007383966, 0.055718475, 0.097449909, 0.133844842, 0.165865385, 0.194255480, 0.219599428, 0.242362525, 0.262919897, 0.281577326, 0.298586572, 0.314156796, 0.328463204, 0.341653666, 0.353853854, 0.365171249, 0.375698324, 0.385515070, 0.394691036, 0.403286979, 0.411356209, 0.418945700, 0.426096998, 0.432846988, 0.439228530, 0.445270988, 0.451000690, 0.456441305, 0.461614173, 0.466538584, 0.471232020, 0.475710357, 0.479988052, 0.484078294, 0.487993139, 0.491743632, 0.495339913, 0.498791297, 0.502106371, 0.505293055, 0.508358663, 0.511309967, 0.514153246, 0.516894321, 0.519538606, 0.522091141, 0.524556617, 0.526939414, 0.529243624, 0.531473069, 0.533631332, 0.535721769, 0.537747525, 0.539711558, 0.541616647, 0.543465405, 0.545260295, 0.547003638, 0.548697622, 0.550344314, 0.551945668, 0.553503531, 0.555019650, 0.556495682, 0.557933194, 0.559333677, 0.560698542, 0.562029131, 0.563326719, 0.564592520, 0.565827686, 0.567033317, 0.568210460, 0.569360112, 0.570483225, 0.571580709, 0.572653430, 0.573702216, 0.574727861, 0.575731122, 0.576712723, 0.577673359, 0.578613694, 0.579534365, 0.580435983, 0.581319132, 0.582184374, 0.583032250, 0.583863275, 0.584677948, 0.585476747, 0.586260131, 0.587028542, 0.587782406, 0.588522131, 0.589248111, 0.589960727)
- *y*range = *c*(0, 1)
- Plot (DD1, PP1, type = “*h*”, col = 4, main = expression (paste (alpha, “ = 0.2”)), cex.main = 1.0, *x*lab = “*x*”, *y*lab = “*h*(*x*)”, lwd = 1, pch = 5)
- Points (DD1, PP1, col = 0); abline (*h* = 26, col = 2)
- Par (new = TRUE)
- Plot (DD1, PP1, type = “*p*”, col = 2, main = expression (paste (alpha, “ = 0.2”)), cex.main = 1.0, *x*lab = “*x*”, *y*lab = “*h*(*x*)”, lwd = 1, pch = 1)
- Par (new = TRUE)
- Estimation code for data set I:
- rm (list = ls())
- Library (fitdistrplus); library (MASS); library (stats 4)
- Data <- *c*(rep(0, 43), rep(1, 35), rep(2, 17), rep(3, 11), rep(4, 5), rep(5, 4), rep(6, 1), rep(7, 2), rep(8, 2))
- ### Write the PMF of your Distribution #################
- dPXL <- function (*x*, alpha) ((alpha^2)*∗*(*x* + 3*∗*alpha + (alpha^2) + 3))/(1 + alpha)^(4 + *x*)
- ### Write the CDF of your Distribution ##################
- pPXL <- function (*q*, alpha)
- 1 − ((1/(alpha + 1)^(4 + *q*)) *∗*(1 + alpha*∗*(*q* + 4 + alpha*∗*(alpha + 3))))
- *f*1 <- fitdist(data, “PXL”, start = list(alpha = 0.86608), discrete = TRUE)
- Summary (*f*1)
- Estimation code for data set II:
- rm (list = ls())
- Library (fitdistrplus); library (MASS); library (stats 4)
- Data < - *c*(rep(0, 200), rep(1, 57), rep(2, 30), rep(3, 7), rep(4, 6))
- ### Write the PMF of your Distribution ##################
- dPXL <- function (*x*, alpha) ((alpha^2)*∗*(*x* + 3*∗*alpha + (alpha^2) + 3))/(1 + alpha)^(4 + *x*)
- ### Write the CDF of your Distribution ##################
- pPXL <- function (*q*, alpha)
- 1 − ((1/(alpha + 1)^(4 + *q*)) *∗*(1 + alpha*∗*(*q* + 4 + alpha*∗*(alpha + 3))))
- *f*1 <- fitdist (data, “PXL”, start = list(alpha = 0.86608), discrete = TRUE)
- Summary (*f*1)
